# Assessment of Structural, Optical, and Antibacterial Properties of Green Sn(Fe : Ni)O_2_ Nanoparticles Synthesized Using *Azadirachta indica* Leaf Extract

**DOI:** 10.1155/2023/5494592

**Published:** 2023-02-07

**Authors:** Abeer S. Aloufi

**Affiliations:** Department of Biology, College of Science, Princess Nourah bint Abdulrahman University, P.O. Box 84428, Riyadh 11671, Saudi Arabia

## Abstract

Metal oxide nanoparticles have attained notable recognition due to their interesting physicochemical properties. Although these nanoparticles can be synthesized using a variety of approaches, the biological method involving plant extracts is preferred since it provides a simple, uncomplicated, ecologically friendly, efficient, rapid, and economical way for synthesis. In this study, the *Azadirachta indica* leaf extract was used as a reducing agent, and a green process was used to synthesize tin(ferrous: nickel)dioxide (Sn(Fe : Ni)O_2_) nanoparticles. The synthesized nanoparticles were subjected to characterization by using X-ray diffraction (XRD), energy-dispersive X-ray (EDX) spectroscopy analysis, field emission scanning electron microscopy (FESEM), Fourier transform infrared (FTIR) spectroscopy, dynamic light scattering (DLS), and photoluminescence (PL) measurement. Furthermore, Sn(Fe : Ni)O_2_ nanoparticles were analyzed for their antimicrobial activity against Gram-positive and Gram-negative organisms including *Staphylococcus aureus, Streptococcus pneumoniae, Bacillus subtilis, Klebsiella pneumoniae, Escherichia coli*, and *Pseudomonas aeruginosa* bacterial strains. XRD patterns revealed that Sn(Fe : Ni)O_2_ nanoparticles exhibited a tetragonal structure. The hydrodynamic diameter of the nanoparticles was 143 nm, as confirmed by the DLS spectrum. The FESEM image showed the spherical form of the synthesized nanoparticles. Chemical composites and mapping analyses were performed through the EDAX spectrum. The Sn–O–Sn and Sn–O stretching bands were 615 cm^−1^ and 550 cm^−1^ in the FTIR spectrum, respectively. Various surface defects of the synthesized Sn(Fe : Ni)O_2_ nanoparticles were identified by photoluminescence spectra. Compared to traditional antibiotics like amoxicillin, the inhibition zone revealed that Sn(Fe : Ni)O_2_ nanoparticles displayed remarkable antibacterial activity against all tested organisms, indicating the valuable potential of nanoparticles in the healthcare industry.

## 1. Introduction

Metal oxide nanoparticles (NPs) differ from bulk materials in terms of their optical, thermal, magnetic, and electrochemical properties [1]. Owing to their small size and distinct features from bulk materials, these are particularly effective in applications such as pharmaceuticals, energy, chemicals, communications, agricultural machinery, manufacturing, industries, and consumer goods [2]. Metal oxide NP characteristics are known to be sensitive to the environment in which they are produced. To synthesize nanoparticles, researchers have employed the hydrothermal approach [3], combustion [4], coprecipitation [5], the sol-gel method [6], and the green method [7]. Due to the utilization of hazardous and harmful compounds, some NP synthesis pathways [8, 9] using ionic liquids, pulsed laser [10], thermal decomposition [11], irradiation through microwaves [12], and so on, are not suitable for the safe fabrication of nanoparticles. As a result, in the field of nanoscience, a green method for synthesizing nanoparticles that are environmentally acceptable, harmless, and inexpensive is required.

Among the various routes of NP synthesis, the green method has some advantages over physical-chemical methods, such as the usage of safe compounds, the ability to synthesize nanoparticles without producing harmful by-products, the lack of toxic reagents, and the fact that it is an environmentally friendly, safe, and low-cost method. Plant extracts serve as both reducing and capping agents [13–15], and the extracts' phytochemicals help decrease and stabilize nanoparticles.

The biological activity of inorganic nanoparticles is influenced by various factors, including their size, morphology, surface charge, surface chemistry, capping agents, and other properties. With regard to the synthesis of NPs, the capping agent is one of the most significant elements. As a result, selecting suitable capping components is critical for stabilizing colloidal solutions as well as their absorption into living cells and the environment. After capping with biocompatible surfactants, the surface chemistry and particle size of nanoparticles are changed. Capping agents should have the ability to decompose and be well scattered, soluble, biocompatible, and nontoxic.

In this regard, for the synthesis of nanoparticles, the *Azadirachta indica* leaf extract was utilized. *Azadirachta indica* (family Meliaceae) is a plant that can be found in abundance across the tropics of the world. It has been shown that *A. indica* leaves possess anti-inflammatory, antipyretic, antimicrobial, antidiabetic, and diverse pharmacological properties [16] by increasing insulin secretion and lowering blood glucose levels. In Asia, the leaves of the plant *(A. indica*) have long been utilized for medicinal purposes. *A. indica* can also be employed as a capping and reducing agent in the manufacturing process of nanoparticles [17].

Semiconductor nanostructures are currently attracting a lot of attention due to their unique physicochemical properties. The N-type semiconductor, SnO_2_ (nanostructured tin dioxide), with a bandgap width of nearly 3.6 eV, has a wide range of applications. SnO_2_ also possesses excellent optical and electrical properties, making it suitable for photocatalysis, solar cells, gas sensors, transistors, and transparent electrodes, and displays high antibacterial activity [18–23].

The doping of SnO_2_ nanoparticles with transition metals or nonmetals has been observed to enhance their physical, chemical, and biological properties. Iron (Fe) is the most popular metal because of its half-filled electronic arrangement, which is expected to aid in narrowing the bandgap by forming new intermediate band levels and trapping electrons to reduce the recombination rate of pairs by catching photogenerated electron/hole pairs [24]. Therefore, a decrease in the recombination consequences of charge carriers is an explanation for how bandgap energy enhances the physical and biological activities of SnO_2_ [25].

The material's structure, surface morphology, composition, optical properties, photocatalytic dye degradation, and antibacterial properties are all thoroughly examined [26]. Previous studies reported that increasing the concentration of Fe-doped ions improved photocatalytic degradation efficiency and antibacterial activity [27]. Particularly, metal and metal oxide NPs are thought to have antibacterial activity due to the generation of reactive oxygen species such as H_2_O_2_, superoxide, and hydroxyl radicals. Reactive oxygen species penetrate the bacterial cell membrane, causing DNA and protein damage and inhibiting bacterial growth [28]. According to XRD and FESEM analysis, the increased antibacterial activity of Fe-SnO_2_ NPs can be attributed to their small particle size, which causes bacterial cells to leak intracellular components and die as a result of reactive oxygen species generated on their surfaces [29].

In the present work, the synthesis of Sn(Fe : Ni)O_2_ nanoparticles was carried out by the green process using the *Azadirachta indica* leaf extract. Structural, morphological, optical, and antibacterial studies were carried out in an attempt to assess their potential to be employed in further biomedical applications.

## 2. Materials and Methods

### 2.1. Materials

Chemicals such as ferrous nitrate nonahydrate (Fe(NO_3_)_3_ ·9H_2_O), tin(II) chloride (SnCl_2_), and nickel(II) nitrate hexahydrate (Ni(NO_3_)_2_·6 H_2_O) were procured from Sigma Aldrich, USA. All other required reagents and chemicals obtained were of high analytical grade.

### 2.2. Preparation of Green Sn(Fe : Ni)O_2_ Nanoparticles

The synthesis of Sn(Fe : Ni)O_2_ nanoparticles by the green method and antimicrobial activity of the entire study are schematically represented in Figure 1.

The freshly collected *Azadirachta indica* leaves were washed multiple times with deionized water to remove adhering foreign impurities. The aqueous leaf extract was prepared by boiling 10 g of fresh leaves at 80°C in 100 ml of deionized water for 15 min. Furthermore, the leaf extract was filtered using filter paper.

First, 0.002 M of ferrous nitrate solution and 0.002 M of nickel nitrate solution were added to an aqueous tin chloride solution (0.096 M). Then, the obtained metal ion solution was mixed with 100 mL of the *Azadirachta indica* leaf extract and magnetically stirred at room temperature for 20 min to achieve a green-colored homogeneous solution. Next, the resultant solution was irradiated by using a microwave at 800 W for 10 min in polypropylene-capped autoclave bottles. Later, the obtained precipitate was cooled to room temperature and washed several times with deionized water and ethanol. At 120°C, the obtained residue was dried, and a light white powder was obtained. Finally, Sn(Fe : Ni)O_2_ nanoparticles were annealed at 800°C for 5 h and then utilized for further analysis.

### 2.3. Characterization of Sn(Fe : Ni)O_2_ Nanoparticles

An X-ray diffractometer (PANalytical X'Pert Pro) was used to characterize the synthesized SnO_2_ and Sn(Fe : Ni)O_2_ nanoparticles. Their morphology and chemical composition were examined by using Carl Zeiss Ultra 55 FESEM with Inca : EDAX). The particle size was used to measure dynamic light scattering (DLS) using NanoPlus instruments. The Fourier transform infrared spectra were measured in the range between 400 and 4000 cm^−1^ by using a Perkin-Elmer spectrometer. The photoluminescence spectra were measured using a JASCO FP-8200 spectrofluorometer.

### 2.4. Antibacterial Activity of Sn(Fe : Ni)O_2_ Nanoparticles

A culture collection from ATCC was used in this study, and using Mueller–Hinton agar (MHA), we tested the antibacterial activity of Sn(Fe : Ni)O_2_ nanoparticles against Gram-positive and Gram-negative bacteria including *Staphylococcus aureus, Streptococcus pneumoniae, Bacillus subtilis, Klebsiella pneumoniae, Escherichia coli,* and *Pseudomonas aeruginosa* based on the Clinical and Laboratory Standards Institute methodology. The nanoparticles were tested at a concentration of 1, 1.5, and 2 mg/ml dispersed in dimethyl sulphoxide (DMSO). The zone of inhibition was measured after incubating the plates at 37°C for 24 h. The antibiotic (amoxicillin) (10 µg disc) was used as a positive control.

### 2.5. Statistical Analysis

The mean and standard deviation of each result were calculated using descriptive statistics. The significant differences between control and treated groups were determined by using Student's *t*-test. *p* value of less than 0.05 was considered significant. SPSS statistical software version 11 (SPSS Inc., Chicago, USA) was employed to perform all statistical analyses.

## 3. Results and Discussion

### 3.1. X-Ray Diffraction (XRD) Analysis

The powder XRD patterns of the synthesized SnO_2_ and Sn(Fe : Ni)O_2_ nanoparticles are shown in Figure 2(a). The diffraction peaks were indexed at 2 *θ* = 26.05°and 26.08° for (1 1 0), 33.31° and 33.36° for (1 0 1), 37.42° and 37.45° for (2 0 0), 51.21° and 51.25° for (2 1 1), 54.21° and 54.25° for (2 2 0), 57.34° and 57.32° for (0 0 2), 61.36° and 61.36° for (3 1 0), 64.22° and 64.23° for (1 1 2), 65.37° and 65.44° for (3 0 1), 70.71° and 70.731° for (2 0 2), and 78.20° and 78.18° for (3 2 1). SnO_2_ and Sn(Fe : Ni)O_2_ nanoparticles exhibit a rutile phase with space group P42/mnm and are well matched to the bulk SnO_2_ standard values (JCPDS card no. 41–1445) [30]. In addition, no secondary phase was observed in the XRD diffraction peaks of Sn(Fe : Ni)O_2_ nanoparticles. This implies that Fe and Ni ions can fit into the lattice sites of SnO_2_ instead of the interstitial space.  Figure 2(b) shows information about the diffraction angle shift in the (1 1 0) hkl plane, which is a shift towards the higher angle side with the substitution of Fe and Ni atoms in the SnO2 surface matrix. These effects are accompanied by changes in lattice parameter values. Debye–Scherrer's equation [31] was used to calculate the average crystallite size of SnO_2_ and Sn(Fe : Ni)O_2_ nanoparticles as follows:

(1) $$\begin{array}{c} average\;crystallite\;size\left(D\right)=\frac{0.9\;\lambda }{\beta \;\cos\;\theta }\text{,} \end{array}$$

where *λ* is equal to 1.54060 Å (the wavelength of X-ray used), *β* is the angular peak width at half maximum in radians, and *θ* is Bragg' s diffraction angle. The average crystallite size is calculated at 65 nm and 52 nm for SnO_2_ and Sn(Fe : Ni)O_2_ nanoparticles, respectively.

### 3.2. Energy-Dispersive X-Ray (EDX) Spectroscopy Analysis

The energy-dispersive X-ray (EDX) spectroscopy spectrum shows the chemical composition of Sn(Fe : Ni)O_2_ nanoparticles, as depicted in Figure 3. In the present investigation, the Sn(Fe : Ni)O_2_ sample only showed the presence of Fe, Ni, Sn, and O elements. However, the EDX image clearly displayed that Fe and Ni ions were successfully substituted into the host SnO_2_ surface matrix. The atomic percentage of Fe is 0.77%, that of Ni is 0.74%, that of Sn is 25.81%, and that of O is 72.68%. The EDX mapping analysis of Sn(Fe : Ni)O_2_ nanoparticles is shown in Figure 3. The elemental mapping results also confirm the purity of nanoparticles. In the present investigation, Sn(Fe : Ni)O_2_ nanoparticles only contain O, Fe, Ni, and Sn atoms distributed uniformly throughout the whole area.

### 3.3. FTIR Spectroscopy Analysis

The FTIR spectra of the *A. indica* leaf extract (Figure 4) display the vibration frequency bands at 3407 cm^−1^ (amide groups of proteins and enzymes), 1638 cm^−1^ (N-H amide), 1386 cm^−1^ (O-H in-plane bend), 1103 cm^−1^ (C-O stretching of alcoholic groups), and 644 cm^−1^ (aromatic C-H out-of-plane bending) [32–34]. The FTIR spectra of the synthesized nanoparticles are shown in Figure 4. The O-H stretching and O-H bending were observed at 3441 and 1627 cm^−1^;respectively, asymmetric and symmetric C-H stretching peaks were at 2917 and 2849 cm^−1^, respectively. The antisymmetric Sn–O–Sn and Sn–O stretching peaks appeared at 615 cm^−1^ and 550 cm^−1^, respectively. This result confirmed that the *A. indica* leaf extract's -OH group attaches to metal ions (ferric, nickel, and tin) and forms a coordination compound.

### 3.4. FESEM and TEM Analysis of Sn(Fe : Ni)O_2_ Nanoparticles

The FESEM images of Sn(Fe : Ni)O_2_ nanoparticles are shown in Figures 5(a) and 5(b). The FESEM images with lower and higher (i.e., ×10,000 and ×50,000, respectively) magnifications were captured at the same operating voltage of 5 kV. The prepared Sn(Fe : Ni)O_2_ nanoparticles were well crystallized and formed spherical and agglomerated shapes. These agglomerated shapes may be due to the strong interaction between hydrogen bonds in the precipitate during the green synthesis [35]. The average size of the nanoparticles in the Sn(Fe : Ni)O_2_ sample was estimated to be between 30 nm. The TEM pattern of Sn(Fe : Ni)O_2_ nanoparticles is shown in Figures 5(c) and 5(d). The different sizes of Sn(Fe : Ni)O_2_ nanoparticles were detected by TEM analysis and plotted as a bar chart based on the count versus particle size, as shown in Figure 5(e).

### 3.5. Dynamic Light Scattering (DLS) Spectrum of Sn(Fe : Ni)O_2_ Nanoparticles

The DLS spectrum estimated the particle size distribution of Sn(Fe : Ni)O_2_ nanoparticles, as shown in Figure 6. The DLS analysis indicated that, for the Sn(Fe : Ni)O_2_ nanoparticles synthesized using the aqueous *A. indica* leaf extracts, the hydrodynamic diameter was 143 nm for the nanoparticles.

### 3.6. UV-Visible Spectroscopy

The UV-visible absorption spectrum of Sn(Fe : Ni)O_2_ nanoparticles doped with sodium alginate is depicted in Figure 7. The prominent absorption peak of the Sn(Fe : Ni)O_2_ nanoparticles is at 271 nm. Electrons moved from the valence band to the conduction band as a result.

### 3.7. Photoluminescence (PL) Spectrum of Sn(Fe : Ni)O_2_ Nanoparticles

Figure 8 shows the PL spectrum of the synthesized Sn(Fe : Ni)O_2_ nanoparticles. The exciting wavelength was found to be 325 nm. The spectrum of PL emission was observed in UV emission due to a recombination of electron-hole pairs and in visible emission due to various intrinsic defects in SnO_2_ nanoparticles including V_Sn_, V_O_, O_Sn_, O_i_, and Sn_i_ corresponding to tin vacancies, oxygen vacancies, oxygen antisites, oxygen interstitials, and tin interstitials, respectively [36]. The PL emission values of Sn(Fe : Ni)O_2_ nanoparticles are 366 nm, 395 nm, 417 nm, 442 nm, 467 nm, 484 nm, 503 nm, and 512 nm. The UV (near-band edge (NBE) emission) emission peak was found to be at 366 nm and 395 nm, which is attributed to the radiative recombination of electrons in the conduction band. The violet emission peak at 417 nm, the three blue emission peaks at 442 nm, 467 nm, and 484 nm, and the two peaks at 503 nm and 512 nm correspond to green emission. These emission peaks are caused by oxygen vacancies (O_i_) and tin interstitials (Sn_i_) in the surface defects of Sn(Fe : Ni) O_2_ nanoparticles.

### 3.8. Antibacterial Activity of Sn(Fe : Ni)O_2_ Nanoparticles

The antibacterial activity of Sn(Fe : Ni)O_2_ nanoparticles was tested by the diffusion method against *S. aureus, S. pneumoniae, B. subtilis, K. pneumoniae, E. coli, and P. aeruginosa* bacterial strains. Both Sn(Fe : Ni)O_2_ nanoparticles and amoxicillin exhibited antibacterial activity, and increasing the concentration of nanoparticles also increased the antibacterial activity, as shown in Figures 9 and 10. As a result of adhering to microbial cell surfaces, Sn(Fe : Ni)O_2_ nanoparticles damage the cell membrane and alter transport activity. As a result of interfacing with cellular organelles and biomolecules, Sn(Fe : Ni)O_2_ nanoparticles affect the respective machinery within microbial cells. In microbial cells, Sn(Fe : Ni)O_2_ nanoparticles cause an increase in ROS, causing damage to the cell, and in a cellular signal system, Sn(Fe : Ni)O_2_ nanoparticles induce cell death.

In general, Sn(Fe : Ni)O_2_ NPs have uneven microsurfaces with the surface containing active molecules, which readily adhere to the bacterial wall and cause damage to the cell membrane, resulting in cellular organelle extrusion and bacterial death. The FESEM images of synthesized Sn(Fe : Ni)O_2_ nanoparticles also displayed uneven ridges at their outer surface, which could have led to the potential antibacterial activity in the current study.

In this study, we determined that Sn(Fe : Ni)O_2_ NPs have antibacterial activity against both Gram-positive (*B. subtilis, S. aureus,* and *S. pneumoniae*) and Gram-negative (*E. coli, P. aeruginosa,* and *K. pneumoniae*) bacteria. A wide variety of metal- or metal ion-based NPs engineered from various nanomaterials have been synthesized. The majority of nanomaterials described in recent studies have antibacterial activity that can be attributed to one or more of the following mechanisms: Cell wall/membrane synthesis is inhibited, energy transduction is disrupted, toxic ROS are produced, photocatalysis is inhibited, enzymes are inhibited, and DNA production is reduced [37]. The Sn(Fe : Ni)O_2_ sample's MIC and MBC for inhibiting bacterial growth are 1.2 and 1.5 mg ml^−1^, respectively, (Table 1).

As shown in Figure 10, Sn(Fe : Ni)O_2_ NPs inhibited only *B subtilis*, then *E coli, P aeruginosa*, and *S. aureus*. The generation of reactive oxygen species (ROS) within the microbial cell membrane is a major reason for the increased antimicrobial effect of Sn(Fe : Ni)O_2_ NPs. ROS generate three types of free radicals to increase antimicrobial properties: hydrogen peroxide (H_2_O_2_), superoxide free radicals (O_2_%), and hydroxyl free radicals (OH%) [38]. As a result of ROS production, NPs in hydrogen peroxide penetrate the cell membrane, causing DNA damage and cell death [39]. In pure Sn (Fe : Ni)O_2_ NPs, higher inhibition zones were observed against *B. subtilis* and reduced activities were observed against *S. aureus, E. coli,* and *P. aeruginosa*. Sn (Fe : Ni)O_2_ NPs have much higher activity against *E. coli* than against *S. aureus*, and Gram-negative bacteria deactivate more efficiently than Gram-positive bacteria.

## 4. Conclusion

In conclusion, an eco-friendly method to synthesize Sn(Fe : Ni)O_2_ nanoparticles using the *Azadirachta indica* leaf extract as a reducing agent has been demonstrated in the current study. The XRD patterns of Sn(Fe : Ni)O_2_ nanoparticles exhibited a tetragonal structure. From the FESEM image, the spherical structure of the synthesized nanoparticles was noticed. Chemical composite and mapping analyses were performed through the EDAX spectrum. Various functional groups were identified using the FTIR spectrum. The antibacterial activity of Sn(Fe : Ni)O_2_ nanoparticles was found to be greater than that of conventional antibiotics such as amoxicillin in this study.

## Figures and Tables

**Figure 1:** Schematic and graphical representation of study design and methods.

**Figure 2:** (a) X-ray diffraction patterns and (b) enlarged version XRD peak 110 plane for SnO_2_ and Sn(Fe : Ni)O_2_ nanoparticles.

**Figure 3:** EDAX spectrum and mapping analysis of Sn(Fe : Ni)O_2_ nanoparticles.

**Figure 4:** FTIR spectra of *Azadirachta indica* leaf extract and Sn(Fe : Ni)O_2_ nanoparticles.

**Figure 5:** The electron microscopic characterization of Sn(Fe:Ni)O_2_ nanoparticles. Lower and higher magnification FESEM (a, b) and the TEM image (c, d) of Sn(Fe : Ni)O_2_ nanoparticles. (e) The histogram TEM image of Sn(Fe : Ni)O_2_ nanoparticles.

**Figure 6:** DLS spectrum of Sn(Fe : Ni)O_2_ nanoparticles.

**Figure 7:** UV-Vis spectrum of Sn(Fe : Ni)O_2_ nanoparticles.

**Figure 8:** PL spectrum of Sn(Fe : Ni)O_2_ nanoparticles.

**Figure 9:** Antibacterial activity of Sn(Fe : Ni)O_2_ nanoparticles.

**Figure 10:** The zone of inhibition of synthesized Sn(Fe : Ni)O_2_ nanoparticles for *S. aureus, S. pneumoniae, B. subtilis, K. pneumoniae, E. coli, and P. aeruginosa* bacterial strains. ^*∗∗∗*^indicates *P* < 0.0005 compared with the control drug; ^*∗∗*^indicates *P* < 0.005 compared with the control drug; ^*∗*^indicates *P* < 0.05 compared with the control drug.

**Table 1:** Determination of MIC and MBC against test pathogens for Sn(Fe : Ni)O_2_ NPs.

Concentration of Sn(Fe : Ni)O_2_(ng ml^−1^)	Effect of Sn(Fe : Ni)O_2_ on the bacterial strains	
	*S. aureus*	*E. coli*
300	Growth	Growth
600	Growth	Growth
900	Growth	Growth
1200	Bacteriostatic (MIC)	Bacteriostatic (MIC)
1500	Bactericidal (MBC)	Bactericidal (MBC)
2000	Bactericidal (MBC)	Bactericidal (MBC)

## Data Availability

All the data incorporated in the manuscript can be obtained from the corresponding author upon request.
